# Exploring the Clinical Point Selection Rules of Acupuncture and Moxibustion in the Treatment of Infantile Enuresis Based on Data Mining Technology

**DOI:** 10.1155/2022/7928052

**Published:** 2022-04-27

**Authors:** Cuicui Ma, Nan Li, Xu Zhang

**Affiliations:** Shijiazhuang Maternity and Child Healthcare Hospital, Shijiazhuang, Hebei 050000, China

## Abstract

In order to explore the clinical point selection rules of acupuncture and moxibustion in the treatment of infantile enuresis based on data mining technology, first, it introduces the principle of data mining technology, the global optimization strategy of information extraction + genetic search. In China Biomedical Literature Database, CNKI, Weipu, Wanfang. Use “enuresis,” “enuresis,” “leathering,” “urinary discharge,” “drowning,” “bedwetting,” “nocturia,” “drowning,” “moxibustion,” “moxibustion,” and “moxibustion” as search terms, take (enuresis + enuresis + urination + urination + addiction + bedwetting), (moxibustion + moxibustion + moxibustion)” as the retrieval style. The analysis of the use of moxibustion, the law of acupoint selection by different moxibustion methods, and the frequency analysis of meridian use show that most of the moxibustion methods are used (62 articles, of which 3 articles use 2 moxibustion methods), including non-suppurative moxibustion, ginger moxibustion, medicinal cake moxibustion, salt moxibustion, mild moxibustion, warm acupuncture moxibustion, bird pecking moxibustion, circling moxibustion, and warm moxibustion; among them, mild moxibustion has the highest frequency of use 24 and non-suppurative moxibustion and salt-separated moxibustion have the lowest frequency of use1; there are 4 non-moxibustion methods, which are medicated thread moxibustion methods. Different moxibustion methods for acupoint selection have their own emphasis. The 63 included literatures included 63 prescriptions for moxibustion, 11 prescriptions for acupoints. Analyzing the frequency of acupoint selection, a total of 18 ear acupoints are involved, and the total frequency of auricular acupoints is 54 times; 44 points are involved (including 1 odd point outside the meridian), the total frequency of acupoints is 300 times, and the total frequency of meridian points is 298, and the total frequency of Jingwaiqi acupoints (Sishencong) is 2. The results can provide great help for the clinical selection of acupuncture points for the treatment of infantile enuresis.

## 1. Introduction

The Pediatric Enuresis Treatment Association (1CCS) defines pediatric enuresis in this way, in children over 5 years of age, intermittent urinary control disorders occur during prolonged sleep at night. However, there is no consensus on the number of times to diagnose enuresis in children; However, in the survey, this standard is about once or more a month [1]. Enuresis is divided into the following four categories: primary, secondary, simple, and complex. The specific situation of secondary enuresis is that the child has been in intermittent urinary incontinence within 6 months of infancy; simple enuresis is after a bed-wetting period of more than 6 months, recurring urinary incontinence, and other situations [2]. Among these categories, children with enuresis are mostly primary simple enuresis. In response to this research question, Grevitt, M. found that children with normal family conditions have a significantly lower incidence of enuresis in children than children from abnormal families. So in social life, for example, the communicative relationship with classmates in school and the punishment of teachers, there are also fierce quarrels caused by the discord between the parents, or it may be due to poor parental management that children watch movies and TV shows that are not suitable for children. Although psychological factors are not directly related to pediatric enuresis, they are of great significance in terms of prevention [3]. Lee, S. H. and Lim, S. believe that children with enuresis are mostly functional disorders, organic diseases do not account for a significant part of this disease, and organic disease is easy to find the cause, so it is not difficult to diagnose [4]. Chen, Q. and others believe that Western medicine has a very deep interpretation and understanding of the etiology and pathogenesis of children with enuresis, most of them are hypotheses that fail to achieve a unified understanding, so they are still in an embarrassing position in the treatment of the symptoms and not the root cause. However, in the treatment, the combination of Chinese and Western medicine should be used to treat children with enuresis, and the effect will be better [5]. At present, the clinical treatment of pediatric enuresis patients in need of medical treatment is still based on drugs, although traditional Chinese medicine has unique advantages in the treatment of children with enuresis; however, the decoction process of the drugs is relatively cumbersome, the high price and inconvenience of taking. Therefore, the study of non-drug treatments with less side effects is the main research direction and focus of current medical workers [6]. As a “green therapy,” acupuncture has abandoned the disadvantages of drug treatment, it has the characteristics of safety, simplicity, effectiveness, and low price, and it has been widely used to treat enuresis in children. On the basis of current research, this topic is aimed at the disease of pediatric enuresis, a comprehensive collection and sorting of prescriptions for acupuncture and moxibustion in the treatment of infantile enuresis in recent literature, through information collection and data mining technology, analyze the acupuncture points and compatibility used in the treatment of infantile enuresis, sort out the frequency of use of acupoints and related characteristics and meridians, create a spectrum of optimal acupoints for children with enuresis, and provide theoretical support for the selection and application of acupoints for the clinical treatment of pediatric enuresis [7].

## 2. Method

### 2.1. Proposal of the Basic Principles

#### 2.1.1. Simple Genetic Algorithm (or Serial Genetic Algorithm)

GAs realize the transfer of relevant knowledge in the search process in a special form of 0/1; this allows it to be well applied in graph theory and combinatorial mathematics with 0/1 code as the result, the difficulty of genetic algorithm for global optimization problems lies in: selection of hybridization probability *p*_*c*_ and mutation probability p_*m*_; the size of the group; encoding method and encoding length; how to control the convergence rate of several individuals in a group. If the convergence rate is too fast, the search process will fall into a local extreme trap, make the search process converge prematurely, and the phenomenon of “premature maturity” occurs; if the convergence speed is too slow, the search process degenerates into the traditional genetic algorithm of Monte-Carlo stochastic simulation process, genetic operations such as hybridization and mutation play an important role in the global traversal of the search process, people usually ignore the promotion of the traversal of feasible domains by the diversity of the population, and this results in blind and repetitive search [8].

### 2.2. Introduction of Data Mining Technology

In the basic operations of genetic algorithm initialization, hybridization, mutation, etc., people mostly realize the assignment of samples in a random way, identify the individuals involved in the cross and the location of the cross, the essence of the genetic optimization process of selecting the individuals to be mutated and the mutation position is the optimal allocation of samples in the search space of the Markov chain stability process based on the Bayesian optimal estimation principle, and it will greatly promote the stability of the Markov chain [9]. In order to realize the characterization of the search space by the sample, use the system information brought by individuals with higher fitness function values for further data mining, and make the genetic process search along the “pseudo-gradient” direction, the author combines the information extraction technology with the sampling rules in the SA method, improve the algorithm's ability to search and traverse the feasible region and the stability of the global optimal solution. The main principle of this method:

1. It is the formation of the individual to enable the individual to effectively extract the effective information in the search space *R*^*s*^, people often use random methods to generate larger samples, realize the characterization of *R*^*s*^. This method is feasible to deal with the process synthesis problem in low-dimensional space, for the process synthesis problem in high-dimensional space, it is reluctant. In process system engineering, most of the comprehensive problems that people encounter are in multi-dimensional space, multivariate NLP (MINLP) problems with knowledge and experience constraints. A large number of rigid, high-order nonlinear constraints make the feasible region of the problem small, usually only occupies a small part of the variable value space. In order to enable the small sample set to fully express the effective information in the search space, avoid the generation of invalid individuals or repeated sampling of *R*^*s*^, use the regular method to extract information in A [10].
2. Mutation operation

Mutation operation is the main component of GAs; it provides the possibility for the algorithm to jump out of the local trap and realize the global traversal under the premise of ensuring the algorithm's global traversal, combine deterministic GAs with information extraction technology to realize data mining in search space.

### 2.3. Global Optimization Strategy of Information Extraction + Genetic Search

Under the condition of a small sample, in order to realize the effective solution of multivariate problems, the following solution strategies are adopted:

1. In the search space, use information extraction technology to generate the initial individual set *po*int_*m*_^*d*^
2. for(*i* = 0; *i* < *m*; *i*++)

Centered on *po*int^*d*^[*i*], *R*[*i*] is the radius to construct the subspace *SubS*^*d*^[*i*] in *S*^*d*^. In *SubS*^*d*^[*i*], a genetic algorithm based on information extraction technology is used to conduct sufficient data mining. Mark the final result of the search as $Best\underline{}Generation\left[i\right]$.

Due to the limitations of mutation and hybridization operations, traditional GAs often fall into local extremes. It is unscientific to simply regard $\left\{Best\underline{}Generation\left[i\right]\left|i=1,\cdots ,\left.m\right\}\right.\right.$ as the final result of global optimization.

In order to prevent “population premature” and improve the search ability to jump out of the local extreme value trap, when the population steadily gathers in a certain area in some way, it can be considered that the system has obtained a credible global extremum solution. The generation of the information space depends on the information extraction of the search space by the initial samples. At the same time, in order to avoid the multi-peak and singularity of the objective function from causing the system to fall into a local extremum, a certain degree of information association and refinement are needed for the search results of the parallel information space. According to the characteristics of small sample information extraction, use knowledge association methods to exchange and associate information between parallel information spaces, provide guarantee for further data mining.

Specific steps are as follows:

Select *n*_*t*_ samples in *R*^*s*^, its point set is *p*_*n*_*t*__^(*t*)^, if *n*_*t*_ is big enough, the point where the optimal value of the objective function on *p*_*n*_*t*__^(*t*)^ should approach the global optimal value *M*.*P*_*n*_*t*__^(*t*)^ can maximize the effective information in *R*^*s*^ under the condition of satisfying i, *i*, *d*.

Step 0: Let *t* = 0, *R*^*s*^ ∈ *R*^*s*,0^, and make *x*^(−1)^ = {*ϕ*}.

Step 1: The system information extraction technology is used to generate a point set *p*_*n*_*t*__^(*t*)^ with *n*_*t*_ points on *R*^*s*,*t*^. Take the point in *p*_*n*_*t*__^(*t*)^ as the information center, construct the search subspace, perform deterministic and regular search for real GAs, and get the feasible solution set *X*_*n*_*t*__.

Step 2: Find *x*^(*t*)^ ∈ *X*_*n*_*t*__ ∪ *x*^(*t* − 1)^ and *M*^(*t*)^ such that *M*^(*t*)^ = *f*(*x*^(*t*)^) ≥ *f*(*y*), ∀*y* ∈ *X*_*n*_*t*__ ∪ *x*^(*t* − 1)^ here: *x*^(*t* − 1)^ = {*ϕ*} is the empty set; *x*^(*t*)^ and *M*^(*t*)^ are currently the best approximations of *x*^∗^ and *M*.

Step 3: Stop criteria: Let *r*^(*t*)^ = {r_1_^(*t*)^, ⋯, r_*s*_^(*t*)^}, r_*i*_^(*t*)^ be the radius of the search subspace. If max*r*^(*t*)^ = max(*r*_1_^(*t*)^, ⋯, *r*_*s*_^(*t*)^) < *δ*, here *δ* is a predetermined small positive number, then *R*^*s*,*t*^ is small enough, *x*^(*t*)^ and *M*^(*t*)^ are accepted as approximate solutions, stop calculation. If max*r*^(*t*)^ ≥ *δ*8, go to the next step.

Step 4: Information association and exchange between different information spaces, in view of the small sample estimation characteristics of information extraction technology, the evolution result in the parallel search space is actually a noisy system output. Under inaccurate system output conditions, in order to avoid falling into the local extremum formed by the multi-peak and singularity of the function, improve search efficiency, adopt association rules based on deterministic information, and realize the exchange of information between different search spaces, in order to determine the information space for further searches.

Step 5: Take *x*^(*t*)^ as the center and max*r*^(*t*)^ as the radius, define a new search space *R*^s,*t*+1^ with a certain space shrinkage ratio, and return to step 1.

### 2.4. Information

China Biomedical Literature Database, CNKI, Weipu, Wanfang. Use “enuresis,” “enuresis,” “leathering,” “urinary discharge,” “drowning,” “bedwetting,” “nocturia,” “drowning,” “moxibustion,” “moxibustion,” and “moxibustion” as search terms, take (enuresis + enuresis + wetting + urination + addiction + bedwetting), (moxibustion + moxibustion + moxibustion) as the search formula [11].

### 2.5. Inclusion Criteria

1. The document type is clinical randomized controlled or semi-randomized controlled trial
2. The research subject was clearly diagnosed as enuresis; the diagnosis and efficacy evaluation system adopted are all recognized standards in China, such as the 1998 International Child Continence Society (ICCS) diagnostic criteria
3. Mainly moxibustion therapy, with clear moxibustion prescription and definite curative effect

### 2.6. Data Extraction

Screen strictly according to the literature inclusion and exclusion criteria, if the literature involves syndrome differentiation and acupuncture points, it will be handled as 1 syndrome type and 1 prescription. Design documentation information extraction table, after the data is entered and saved, it is extracted and sorted. The data entry process was completed independently by two people and the consistency check was carried out.

## 3. Results and Analysis

### 3.1. Analysis of the Use of Moxibustion and Analysis of Acupoint Selection Rules of Different Moxibustion Methods

A total of 2528 articles were retrieved in this research; finally, a total of 63 articles were included. Analysis of the use of moxibustion found that moxibustion is mostly (62 articles, there are 3 articles using 2 kinds of moxibustion) including non-suppurative moxibustion, ginger moxibustion, medicinal cake moxibustion, salt moxibustion, mild moxibustion, warm acupuncture moxibustion, bird pecking moxibustion, circling moxibustion, and warm moxibustion; among them, mild moxibustion has the highest frequency of use 24 and non-suppurative moxibustion and salt-separated moxibustion have the lowest frequency of use1; there are 4 non-moxibustion methods, which are medicated thread moxibustion methods. Different moxibustion methods on acupoint selection have their own emphasis on acupuncture points [12]. See Table 1 for details.

### 3.2. Analysis of Frequency of Meridian Use

A total of 11 meridians are involved; the distribution of meridians is shown in Table 2. The meridian acupoints used are mainly concentrated in the Ren Channel and Zutaiyang Bladder Channel [13]. The acupoints belonging to Ren Mai shared 104 times, the acupoints belonging to the full sun bladder meridian share 73 times, the acupoints of the two meridians were used 177 times in total, accounted for 66.0% of the total frequency, and a total of 19 acupoints are used, accounting for 50.0% of the meridian acupoints used.

### 3.3. Analysis of Acupoints in the Treatment of Enuresis by Moxibustion

The 63 included literatures included 63 prescriptions for moxibustion, 11 prescriptions for acupoints. Analyze the frequency of acupoint selection, involving 18 ear acupoints, the total frequency of ear points is 54 times; 44 acupoints are involved (including 1 acupuncture point outside the meridian), and the total frequency of acupoints is 300 times, the total frequency of meridian points is 298, and the total frequency of meridian acupoints (Sishencong) is 2 [14]. Arrange the ear acupoints with the top 9 frequency of use and the 12 acupoints with the top 12 frequency of use in descending order. See Table 3 and Figure 1 for details.

Regarding NE, different countries have different diagnostic standards, the main difference is the frequency of enuresis and age. According to the definition established by the International Children's Continence Association in 2006, NE is age>5 years old, children without central nervous system disease, involuntary leakage of urine during sleep, at least twice a week for ≥3 months. According to different performance characteristics, enuresis is divided into single symptom nocturnal enuresis and compound symptom nocturnal enuresis; the enuresis discussed in this article is a kind of single-symptomatic nocturnal enuresis, refers to enuresis in which symptoms persist since childhood (the asymptomatic period does not exceed 6 months); it is representative and frequently occurs in clinical practice. Enuresis in Chinese medicine belongs to the category of “drowning,” drowning was first seen in the “Internal Classics”; this name is still used in the “A-B Classic of Acupuncture and Moxibustion”, or it is called enuresis, wetness, and urination [15]. The physician Wanquan of the Ming Dynasty believed that the physiological and pathological characteristics of children were more than two, “three deficiencies”; the liver often has surplus, and the spleen is often insufficient; the heart is often surplus, and the lungs are often insufficient; the kidney is often weak, and the lack of the lung, spleen, and kidney is more prominent. Children with enuresis are mostly with deficiency syndrome 0; therefore, the treatment is based on the principles of invigorating the kidney and cultivating vitality, replenishing qi and invigorating the spleen, the spleen qi can be raised, the lung qi can be lowered, the bladder can be restrained, and enuresis can be stopped. The results of this study suggest that there are many ways to treat enuresis with moxibustion, and the selection of acupoints is spread across many meridians and has obvious regularity; ear acupoints are widely used and the effect is obvious [16].

This study found that moxibustion used suspension moxibustion (including gentle moxibustion, bird pecking moxibustion, and circling moxibustion) in the treatment of enuresis, moxibustion points are based on the acupoints on the lower abdomen (Guanyuan, Qihai, etc.), the lower waist acupoints (Shenshu, Bladdershu, etc.) of the full sun bladder meridian are mainly used, and moxibustion heat can directly penetrate into the related viscera and play a direct therapeutic role. The compatibility of acupoints is an important part of the acupuncture treatment system; it has a direct impact on clinical efficacy. Faced with complex diseases, acupuncture is based on the theory, method, prescription, and acupoint theory of TCM acupuncture and moxibustion, that is, based on the differentiation of meridians and collaterals, guided by viscera differentiation, compatibility of acupoints for the cause and pathogenesis of the disease, a prescription for acupuncture and moxibustion that fits the disease syndrome is proposed for treatment. The analysis of association rules of acupoints shows that the highest support is Yidanshu, Baihui, Shenshu, Zhongji, Guanyuan, and Sanyinjiao. In terms of distribution, the meridian points used in moxibustion treatment of enuresis are mainly concentrated in Ren Channel, foot Taiyang bladder meridian, and foot Taiyin spleen meridian. The three meridians all pass through the trunk. Ren Mai and foot Taiyin spleen meridian connect to the abdomen, and the full sun bladder meridian is connected to the lower back [17]. Guanyuan, Shenshu, Zhongji, and Sanyinjiao, the first three acupoints used frequently, are the points of Ren Mai, Zutaiyang bladder meridian, and foot Taiyin spleen meridian, respectively, that reflect the short-term and far-reaching effects of “the meridians pass through and the main treatment reaches” [18].

## 4. Conclusion

This study found that moxibustion used suspension moxibustion (including mild moxibustion, bird pecking moxibustion, and circling moxibustion) in the treatment of enuresis, moxibustion points are based on the acupoints on the lower abdomen (Guanyuan, Qihai, etc.), the lower waist acupoints (Shenshu, Bladdershu, etc.) of the full sun bladder meridian are mainly used, and moxibustion heat can penetrate directly into the related viscera and play a direct therapeutic role. The compatibility of acupoints is an important part of the acupuncture treatment system; it has a direct impact on clinical efficacy. Faced with complex diseases, acupuncture is based on the theory, method, prescription, and acupoint theory of TCM acupuncture and moxibustion, that is, based on the differentiation of meridians and collaterals, and guided by the differentiation of viscera, compatibility of acupoints for the cause and pathogenesis of the disease, a prescription for acupuncture and moxibustion that fits the disease syndrome is proposed for treatment. The analysis of the association rules of acupoints showed that the highest support was Yidanshu, Baihui, Shenshu, Zhongji, Guanyuan, and Sanyinjiao.

## Figures and Tables

**Figure 1:** Moxibustion treatment of enuresis, the frequency of ear acupoint use, the first 9 acupoints.

**Table 1:** The law of selecting points for different moxibustion treatments for enuresis.

Moxibustion	Classification	Number of documents	The law of acupoint selection
Moxibustion	Non-suppurative moxibustion	1	Foot sun bladder meridian, the main acupoints on the lower waist of the Du Channel (Mingmen, Shenshu, Bladdershu, Guanyuanshu);
	Ginger moxibustion	4	① Ren Mai Zhongji, Guan Yuan is the main; ② the Backshu points (Shenshu, Bladdershu, etc.) of the waist under the foot sun bladder meridian are mainly; ③ Zusanli, the stomach meridian of foot Yangming, foot Taiyin, and spleen meridian Sanyinjiao dominate;
	Medicinal cake moxibustion	8	① Ren Mai Shenque is the master; ② Beishu acupoints (Shenshu, Bladdershu) at the waist under the foot sun bladder meridian are mainly;
	Salt moxibustion	1	Ren Mai Shenque is the master;
	Gentle moxibustion	24	① Ren Mai Zhongji and Guanyuan are the main ones; ② the Backshu points (Shenshu, Bladdershu, etc.) of the waist under the foot sun bladder meridian are mainly; ③ Footyangming stomach meridian Zusanli, foot Taiyin spleen meridian Sanyinjiao dominate, and Zushaoyin kidney meridian are dominated by Yongquan;
	Warm acupuncture	8	① Ren Mai Zhongji and Guanyuan are the main ones; ② foot Taiyin and spleen meridian are mainly Sanyinjiao; ③ the main points of Backshu (Shenshu, Bladdershu) in the lower waist of the full sun bladder meridian; ④ emphasize the selection of acupoints based on syndrome differentiation;
	Pecking moxibustion	5	① Ren Mai Guanyuan points are the main points; ② Beishu acupoints at the waist under the foot sun bladder meridian are the main points;
	Convolute moxibustion	2	① Ren Mai Zhongji, Guanyuan, and Qihai are the main ones; ② foot Taiyin and spleen meridian Sanyinjiao dominate;
	Moxibustion	9	① Ren Mai Zhongji, Guanyuan, and Qihai are the main ones; ② Beishu points (Shenshu, Bladdershu, Sanjiaoshu) at the waist under the foot sun bladder meridian are mainly; ③ Fooyangming stomach meridian Zusanli and Zutaiyin spleen meridian Sanyinjiao are the main ones;

Non-moxibustion	Medicinal thread moxibustion	4	① Governor Channel Baihui is the main one; ② Ren Mai Zhongji and guan yuan are the main ones; ③ Beishu acupoints (Shenshu, etc.) at the waist under the foot sun bladder meridian are mainly; ④ Fooyangming stomach meridian Zusanli, Zutaiyin spleen meridian Sanyinjiao are the main ones;

**Table 2:** Meridian analysis of moxibustion treatment of enuresis.

Meridian	Total frequency of acupoints	Frequency/%	Number of acupoints	Frequency/%
Ren Mai	104	34.9	7	15.9
Bladder Channel	77	26.1	13	29.6
Spleen Channel	33	11.4	2	4.6
Governor vessel	32	10.2	4	9.1
Stomach meridian	21	7.2	3	6.8
Stomach meridian	11	3.4	4	9.1
Heart sutra	4	1.2	1	2.3
Liver Channel	4	1.2	1	2.3
Gallbladder	2	0.7	2	4.6
Lung Channel	3	0.8	2	4.6
Large intestine meridian	2	0.7	2	4.6

**Table 3:** Moxibustion treatment of enuresis, the top 12 acupoints used frequently.

Serial number	Acupoints	Frequency	Frequency
1	Guan yuan	46	74.5
2	Shenshu	31	47.8
3	Middle pole	27	44.3
4	Sanyinjiao	27	44.3
5	Bladdershu	21	32
6	Baihui	18	30
7	Zusanli	18	30
8	Qihai	15	25.2
9	Shenque	11	16
10	Pishu	7	12.5
11	Feishu	6	10.9
12	Yinlingquan	5	9.3

## Data Availability

The data used to support the findings of this study are available from the corresponding author upon request.
